# Visual Information Computing and Processing Model Based on Artificial Neural Network

**DOI:** 10.1155/2022/4713311

**Published:** 2022-09-30

**Authors:** Junling Wang, Shuhan Liu

**Affiliations:** ^1^School of Journalism & Communication, Lanzhou University, Lanzhou, Gansu 730000, China; ^2^School of Information Science and Engineering, Lanzhou University, Lanzhou, Gansu 730000, China

## Abstract

This paper analyzes the parallel and serial information processing structure of visual system and proposes a visual information processing model with three layers: visual receptor layer, visual information conduction and relay layer, and information processing layer of visual information computing and processing area. Based on the analysis, abstraction, and simplification of the biological prototype of each layer in the visual system, a framework model of an artificial neural system corresponding to the visual system is proposed. An artificial neural network model is proposed to simulate the mechanism of visual attention. A network model is formed by introducing the saliency mask map as additional information on the benchmark network, and the selective enhancement operation is performed on the extracted features in different regions according to the mask map. The experimental results show that the visual computing processing network model can effectively improve the classification performance of the network when the appropriate saliency mask is used. The visual information computing and processing model network can work effectively for different data sets and different structures of the benchmark network, which is a universal network model. The complexity of visual information computing and processing model network is very small, and the improvement of network performance is not at the cost of increasing model complexity, but in the way of improving network efficiency. The performance of artificial neural network visual information computation and processing model is directly related to the performance of saliency map used as mask map.

## 1. Introduction

At present, the basic framework of computer vision research is still computational vision theory. The hierarchical idea of this theory holds that a high-level computational problem can be independent of the understanding of the algorithm that performs the computation. Algorithmic problems can be solved independently of the understanding of their physical implementation. This view has already caused controversy. There is a strong objection that the assertion of the independence of the levels confuses two completely different types of problems. The first question is, is it possible to understand algorithms and analytical problems regardless of experimental facts? The answer is clearly no. The second question is, can a given algorithm that performs a task on a given machine be implemented on other machines with different structures? The answer is yes. More than 80% of the external world information acquired by human beings is visual information. Therefore, visual information processing is one of the most deeply studied fields in the whole neuroscience [1]. For how the colorful external world becomes the process of human vision, optic neuroscientists have done a lot of outstanding research work from the retina to the cerebral cortex and made a series of important research results, and these results have laid a solid foundation for the study of visual system models and algorithms.

Under such a development trend, the improvement of the current artificial neural network model has met a bottleneck, and simply increasing the depth of the network could not continue to effectively increase the performance of the network, but put forward high requirements for the computing performance of the computer. Model complexity of ascension will bring training and ability of the model to express the increase of the difficulty, and now has more training speed is close to and exceed the speed limit of model expression ability, lead to the improvement of traditional network structure, improve the network complexity, and use various means to decrease the difficulty of the training is in the bottleneck. In fact, the current research focus has gradually shifted from improving network performance to reducing model complexity and computational load without reducing network performance [2]. Now, it is urgent to develop a new idea to make further improvement of the artificial neural network algorithm. And the human visual attention mechanism can make the human visual system achieve high performance. If the visual attention mechanism is introduced into the artificial neural network model, the performance of the neural network can be improved by a method that does not increase the complexity of the model.

Based on the information transmission and processing mechanism provided by the visual system prototype, this paper proposes a comprehensive artificial neural network model of the visual nervous system by applying the research results of the artificial neural network, computer vision, and artificial intelligence. In order to further study the visual system, we should make full use of the research results of cells and molecules, and combine the advantages and research strategies of different disciplines. We can refer to the visualization system implementation technology of neural mechanism. Therefore, an artificial neural system model based on the neural mechanism of the visual system is proposed in this paper. The implementation of this model can be integrated by various artificial neural networks according to different basic visual information processing needs.

## 2. Related Work

With the enhancement of computing performance, artificial neural networks with more parameters and more complex structure can be put into practical application because the implementation of the artificial neural network on the CPU can accelerate the operation speed to ten times or even tens of times [3], which greatly improves the training speed of the artificial neural network and thus accelerates the development speed of artificial neural network technology. The proposed AlexNet used two graphics cards for training and won the championship of several international competitions with an overwhelming advantage [4], which ushered in the second climax of the development of artificial neural network technology. Another famous cat experiment was also carried out: convolutional neural network was used to automatically identify the concept of the cat from video through unsupervised learning [5]. Subsequently, a large number of researchers have invested in the research of artificial neural network technology and constantly refresh records on public data sets. The proposed convolutional artificial neural network achieves 99.79% correct rate on the handwritten database MNIST (Mixed National Institute of Standards and Technology database), and the proposed multicolumn deep neural network achieves 99.77% correct rate on the MINST. Meanwhile, the best result obtained by using the SVM method on MNIST is only 99.4% [6], and the best result obtained by using the K-nearest neighbor method is only 99.3%. For the first time, the classification error rate on ImageNet is lower than the human classification error rate (5.1%) [7]. In some of the larger scale, the number of images, and more variety of database test results, artificial neural network technology is overwhelming. Since then, after several years of research by a large number of researchers, the structure of artificial neural networks has been developed from several layers, dozens of layers in the early years to hundreds of layers. Models such as A1exNet [8], VGG [9], ResNet [10], DenseNet [11], and DPN (digital packet network) [12] are all classical network models appearing in this development process. In addition to these classical structural improvements, there are also the proposed Dropout and Dropconnect [11] regularization methods and the proposed trainable activation function structure maxout [12]. Due to the deepening of network layers in this stage, the focus of research also began to focus on how to solve the problems of gradient explosion, gradient disappearance, overfitting, and so on caused by the increase of network layers, and the artificial neural network technology in this stage gained the name of deep learning. And now, the research of artificial neural network has fallen into a bottleneck.

A classical problem in computer vision is the recognition of objects in images. There are many different forms of object recognition, such as image classification, detection, and image segmentation [13]. Among them, the main goal of the image classification problem is to judge the category of objects contained in a given image, that is, what the target is. The problem of object detection is further based on the problem of image classification, which not only determines what the object is but also locates the spatial position of each object, that is, where the object is. The goal of the image segmentation problem is to find all the pixels corresponding to each object in the image, so it can be regarded as a classification task for each pixel [14, 15]. These three problems are the classical problems in computer vision object recognition task, and also the basic problems to be solved before the construction of complex vision system, which are of great significance in practical applications. In the face of various challenges in the field of computer vision, researchers have proposed a series of algorithms based on statistical features, which are often referred to as traditional computer vision algorithms. Traditional visual algorithms usually rely on statistical methods to extract features in images, such as HOG [16]. After extracting features, these algorithms usually use traditional machine learning algorithms such as logistic regression to get the final results. For different application scenarios, the statistical laws of features are usually different, so the methods of feature extraction in different visual tasks are often different [17]. Traditional computer vision algorithms have achieved good results in some simple visual tasks, but the results are still not ideal in most visual tasks, and it is difficult to meet the complex requirements of various application scenarios. In the object detection task, CNN-based object detection model-1 can usually be divided into a two-stage detection model [17] and a one-stage side detection model [18].

Generally speaking, the former has a higher detection accuracy, while the latter can achieve a faster detection speed. For example, the proposed MegDet model adopted a two-stage detection framework and achieved 52.5% mmAP in the challenge [19], winning the champion of that year's competition. The proposed Pelee uses a single-stage detection framework and achieves a detection speed of 17fps on the device [19]. The method of designing a special feature extraction network for object detection task is explored, and DetNet is proposed, which can improve the precision of side detection while reducing the computation. In the task of image segmentation, the model based on the full convolutional network [20] has become the mainstream method to solve the problem of semantic segmentation. Among them, a series of models [21] constantly refresh the optimal results of semantic segmentation problems. The proposed GCN model points out the necessity of large convolution kernels and large receptive fields in semantic segmentation tasks [22]. For instance segmentation, the proposed model combines the segmentation model and object detection model in parallel [23] and uses the alignment operation to extract feature I for each candidate target region, which simultaneously improves the accuracy of instance segmentation and object detection. In recent years, the increase in network depth makes the training and optimization of the model increasingly difficult [24–26]. It is difficult to continue to improve the network model by increasing the depth of the network. Therefore, in recent years, the research hotspots in related fields have also begun to change. On the one hand, researchers have begun to study how to simplify the network structure and obtain the maximum performance with the minimum amount of computation while slightly improving or maintaining the network performance. On the other hand, researchers began to study more specific algorithms for data sets combined with more specific application scenarios.

## 3. Prototype and Model of Visual Information Computation and Processing Based on Artificial Neural Network

### 3.1. Artificial Neural Network Model for Biological Prototype of Visual Information Computation and Processing

The visual signals are processed by the neural network of the retina and then transmitted from the optic nerve to the visual center. The visual information is computed and processed after the geniculate body of the lateral thalamus. Complex information processing in the computation and processing of visual information leads to visual perception. The neural cells of visual information computation and processing have a columnar fabric pattern. In addition, as in the retina and the external geniculate body, the computation and processing of visual information in visual information processing show both obvious serial characteristics and obvious parallel characteristics. Based on the regulating effect of the external genu body on the visual information flow, the relay visual information processing link controls the visual information flow from retina to visual information computation and processing in a linear or nonlinear adjustable “valve” manner, which is realized by the modeling scheme shown in Figure 1.

1. Studies on functional architecture of visual information computation and processing show that cells with similar receptive field response characteristics tend to cluster into columnar structures in visual information computation and processing. Therefore, visual information computation and processing are organized as vertical cell populations with similar functional properties.
2. Serial processing of visual information computation and processing: The proposed hierarchical hypothesis holds that, in visual information computation and processing, more complex receptive fields are formed by the orderly synthesis of simpler receptive fields at lower levels of visual information processing. In fact, the receptive field processes motion and color information by adopting serial hierarchical processing in their respective parallel pathways to gradually extract meaningful information.
3. Parallel processing of visual information computation and processing: Numerous studies have shown that the visual system is organized into different pathways to transmit and process different aspects of visual information. From the perspective of parallel information processing, a single cell or cell group does not represent a certain characteristic state at the level of perception but only represents some special aspects of the perceived object. In other words, the separate parts do not represent the whole, but the relationship between them constitutes the perception of the whole.
4. Attention mechanism to realize the interrelation of different parts, the brain must integrate the information processing independently completed in different cortical regions through some mechanism. Research shows that attention must be involved in the process of such synthesis. “Attention” will emphasize the specific properties of an object, highlighting significant visual targets, while ignoring other properties of the object and other objects.

According to the analysis of biological prototype of visual information computation and processing, on the one hand, different visual information attributes are processed separately in different visual areas of visual information computation and processing. On the other hand, there are projections between different visual areas. Feed-forward, feedback, and local connections in visual interval are the basis for visual information computation and processing to integrate various visual information and produce vision.

Based on assumption that neurons function hierarchically, there should be complex cells that can bring together huge visual information. Therefore, several functional clusters realized by neural networks are designed in the artificial visual information computing and processing model, and the integration of various kinds of visual information is completed by various functional clusters. For example, feature clusters that recognize characters, feature clusters that recognize fingerprints, feature clusters that recognize faces, and so on. Neurobiological studies have shown that the cortex is plastic. Therefore, visual information computing and processing must gradually form specific brain regions by adapting their functions to important stimuli. This kind of self-learning, self-organization, and self-adaptability can be realized by neural network training algorithm.

### 3.2. Visual Attention Computational Model Based on Target Characteristics

This paper presents a visual attention computation model based on the characteristics of the target itself, which only uses the target information but does not consider the background information of the target. The model includes training stage and attention stage. In the training stage, the color feature is decomposed into three parts: red, green, and blue. The brightness feature includes darker and brighter, the orientation feature includes four directions, and the texture feature also includes two types. Therefore, there are eleven features in total. Background information extraction depends on the target itself rather than on these features. At the same time, the bottom-up saliency map is obtained by the contrast of the graph to be noticed, and the product of these two saliency maps gives the global saliency map. Finally, the size of each saliency region is obtained by maximizing the entropy method. This model has two contributions. One is that the extracted features only depend on the characteristics of the target itself, but not on the background information. The other one is the global saliency plot which is the point-to-point product of the top-down saliency plot and the bottom-up saliency plot. The experimental results show that the model is superior to the pure bottom-up model. When the target to be noticed does not always appear in the background of the training target, or the combination of the target to be noticed and its background is very different from the combination of the training target and its background, the model in this chapter is superior to the VOCUS top-down model and Navalpakkam model.

In the task of finding a red cup in a given input scene, the main flow of the visual attention model based on the features of the target itself is shown in Figure 2. First, the features of the target are extracted from the training image, and each feature is expressed as the mean and standard deviation. Second, the feature information is used to compare the similarity with the features in the input scene to form a top-down saliency map. Third, according to the characteristics of the input scene itself, the bottom-up saliency map is obtained. Finally, the top-down and bottom-up saliency maps are fused to generate a global saliency map to guide visual attention to the possible location of the target.

Error estimation in visual computing is developed on the basis of image processing. It studies the cognitive process of visual information from the level of information processing and studies the computational theory, expression, and computational methods of visual information processing. Error analysis has been a very difficult and rarely studied problem in all stages of visual information processing. However, there is an obvious drawback that it does not reflect the error characteristics of the structure and distribution, and meaningful subtle differences may lead to wrong decisions. The reliability and stability of the visual algorithm are poor, and the calculation results cannot be estimated sometimes and can only be verified by experiments, which fundamentally limits the generality of the visual algorithm. Therefore, how to establish the corresponding error estimation method in each stage of visual information processing is a field worthy of further study in computer vision. The correct estimation of visual computation error will in turn provide a basis for the improvement of the algorithm. The study of a more refined morphological matching error analysis method can effectively improve the reliability and stability of the 3D morphological estimation algorithm because the morphological matching error analysis is based on the structural characteristics of the error, which is more in line with human perceptual characteristics. As a practical technique, its computation has the characteristics of high efficiency and high parallelism.

The work of the visual attention mechanism can be divided into two different working modes. One is a bottom-up, feature-driven visual saliency mechanism, and the other is a top-down, task-driven selective attention mechanism. For an input visual scene, areas with more distinctive features and stronger contrast usually have higher visual saliency, and these areas with higher visual saliency will attract more attention. So when we look at this image, our attention is drawn to the little girl in the image. Therefore, inspired by the visual attention mechanism, in order to further improve the performance of the computer vision model, we propose a structure that can simulate the feature extraction function of the visual attention mechanism in the convolutional neural network. First of all, in order to simplify this problem, we introduce some prior knowledge: we directly use the existing visual saliency algorithms, calculate and process the input image data according to these existing visual saliency algorithms, and obtain the saliency mask map corresponding to each image. These saliency masks are introduced into the training of convolutional neural networks as prior knowledge. In this way, we solve the problem of how the human visual system obtains the global saliency score of the input visual scene by using the existing saliency algorithm.

The input original feature map usually comes from a convolution connection. Here, we express the formula of convolution connection in a general form:

(1) $$\begin{array}{c} t_{jk}=\sum^{}u_{jk}+x_{jk},\\ x_{jk}=f\left(z_{jk}\right). \end{array}$$

Then, according to the design idea explained above and the connection structure shown in the figure above, we can obtain the forward propagation formula of the connection as follows:

(2) $$\begin{array}{c} z_{jk}=y_{ij}*s_{jk}. \end{array}$$

After obtaining the forward and backward transfer formulas, we can make a preliminary and simple analysis of its working principle. It can be seen from the formula that, during forward propagation, the value of each pixel on the enhanced feature map is obtained by enlarging the value of each pixel on the original feature map in equal proportion to its significant value for the location pixel. So we can determine, in the forward propagation, after dealing with the connection, a significant degree of mask value larger area on the graph, which is considered more important areas, will be multiples of corresponding amplified to a larger area, by contrast, a significant degree of mask graph value smaller areas, which is considered less important area, only corresponding amplification area into smaller multiples. Therefore, in the process of forward propagation to obtain the final classification result, the features from more important regional parts will obviously have a greater impact on the classification result.

This structure can be regarded as a subartificial neural network consisting of only one layer of convolutional connections, through which the saliency mask map is trained. In fact, as long as the final output is a saliency mask map of the same size as the feature map, we can design a convolutional neural network with any structure, take any number of saliency mask maps as input, and use the error information feedback from the connection to train the network. Using such a scheme to obtain the enhanced saliency mask can theoretically make very fine adjustment and optimization of the input saliency mask. Even further, we can no longer need to use the trained saliency mask map as additional input prior knowledge but can design a network for obtaining the saliency mask map directly from the input image. This is shown in Figure 3.

## 4. Example Verification

The top-down visual attention model processes tasks that point to the target of a particular task. There are two types of experiments: one is a known task type, and the synthesized scene belongs to this type. The other is the unknown task type. In this case, the task type to be processed is obtained according to the method in the target representation, and most natural scenes belong to this type.  Figure 4 shows the experimental results of the single-target composite image scene, and all the experimental results of the single-target scene are shown in Figure 4.

Figure 5 shows a more detailed comparison of MENet with these network models. These comparison results prove that MENet has stronger feature representation ability in different application scenarios.

In visual information processing, the real-time performance is critical, so the size of the gateway time delay is an important indicator of success for the gateway, and the gateway created in order to get the time delay, under laboratory conditions, was measured by the gateway in the CAN. Data as shown in Table 1.

The spatial diagram of visual information computation and processing operator of the two-dimensional artificial neural network is shown in Figure 6. With different values, *g*(*x*, *y*) can constitute different bandpass filters. By selecting different receptive field fovea width parameter D, the purpose of extracting different spatial frequency information can be achieved. The visual information calculation and processing operator of artificial neural network has shown good performance in many aspects. The concentric circle antagonistic receptive field of biological optic nerve cells can be described by the visual information computing and processing operator of artificial neural networks.

Although the visual information computation and processing operator of artificial neural network has good performance in many aspects, it has great shortcomings in the extraction of orientation information because the visual information computation and processing operator of artificial neural network is not directional. Especially, in recent years, many biologists have found that biological optic nerve cells have obvious orientation selectivity, and morphological studies have shown that the elongated oval dendrites of optic cells may be the basis of orientation selectivity.

The spatial diagram of the visual information computation and processing operator of artificial neural network is shown in Figure 7. Below, the operation mechanism and characteristics of the visual information computation and processing operator of artificial neural network are analyzed.

In summary, the visual information computation and processing operator of artificial neural networks has two important characteristics: (1) we highlight the characteristics of the central region and suppress the surrounding region and (2) the characteristics of direction selectivity. It is these two characteristics of the operator that enable it to simulate the attention mechanism of the nonclassical receptive field of biological vision and to fully take into account the two important elements of gray level and orientation in the extraction of salient area information in the process of visual bottom-up.

## 5. Conclusion

The visual system has three layers of information processing structure: the visual receptor layer, the visual information conduction and relay layer, and the information processing layer in the visual cortex area. The layers are not independent of each other, and there are numerous couplings and interactions. Our research shows that modeling the brain's visual system in a reasonable manner, in addition to from the angle of computational neuroscience, provides theoretical support for the further study of visual electrophysiology and experiment guidance, will also be in biological vision and set up a bridge between computer vision, and is expected to be as many images as the carrier of the engineering application provides efficient front-end preprocessing solution. Most visual information processing processes are multiinput, nonlinear, and sensitive to errors caused by noise or discretization, so model-based computer vision systems cannot be applied. In the next step, artificial neural network will become an important means to solve such problems with its superior nonlinear pattern classification performance and strong self-organization and self-learning ability.

## Figures and Tables

**Figure 1:** Relay information processing model.

**Figure 2:** Visual attention model based on target characteristics.

**Figure 3:** Training multiple input saliency maps.

**Figure 4:** Experimental results of all single-object scenarios.

**Figure 5:** The MENet model outperforms all the compared network models at all four computational magnitudes.

**Figure 6:** Visual information computation and processing operator spatial diagram of artificial neural network. (a) Visual information computation and processing operator of ON artificial neural network. (b) Visual information computation and processing operator of OFF artificial neural network.

**Figure 7:** Spatial diagram of visual information computation and processing operator of artificial neural network.

**Table 1:** Time delay of CAN standard frame.

Baud rate	1.3 ms	4.7 ms	9.5 ms	19.5 ms
220	65	18	10	6
510	65	16	9	5
755	67	18	8	6

## Data Availability

The data used to support the findings of this study are available from the corresponding author upon request.
